# Heart Disease Prediction Based on the Embedded Feature Selection Method and Deep Neural Network

**DOI:** 10.1155/2021/6260022

**Published:** 2021-09-29

**Authors:** Dengqing Zhang, Yunyi Chen, Yuxuan Chen, Shengyi Ye, Wenyu Cai, Junxue Jiang, Yechuan Xu, Gongfeng Zheng, Ming Chen

**Affiliations:** ^1^Jinjiang Hospital Affiliated to Fujian Medical University, Fujian, Jinjiang 362200, China; ^2^Department of Cardiology, Jinjiang Hospital of Fujian Province, Fujian, Jinjiang 362200, China; ^3^School of Informatics Xiamen University, Xiamen University, Fujian, Xiamen 361000, China; ^4^Department of Public Health, Jinjiang Hospital of Fujian Province, Fujian, Jinjiang 362200, China

## Abstract

In recent decades, heart disease threatens people's health seriously because of its prevalence and high risk of death. Therefore, predicting heart disease through some simple physical indicators obtained from the regular physical examination at an early stage has become a valuable subject. Clinically, it is essential to be sensitive to these indicators related to heart disease to make predictions and provide a reliable basis for further diagnosis. However, the large amount of data makes manual analysis and prediction taxing and arduous. Our research aims to predict heart disease both accurately and quickly through various indicators of the body. In this paper, a novel heart disease prediction model is given. We propose a heart disease prediction algorithm that combines the embedded feature selection method and deep neural networks. This embedded feature selection method is based on the LinearSVC algorithm, using the L1 norm as a penalty item to choose a subset of features significantly associated with heart disease. These features are fed into the deep neural network we built. The weight of the network is initialized with the He initializer to prevent gradient varnishing or explosion so that the predictor can have a better performance. Our model is tested on the heart disease dataset obtained from Kaggle. Some indicators including accuracy, recall, precision, and F1-score are calculated to evaluate the predictor, and the results show that our model achieves 98.56%, 99.35%, 97.84%, and 0.983, respectively, and the average AUC score of the model reaches 0.983, confirming that the method we proposed is efficient and reliable for predicting heart disease.

## 1. Introduction

Heart disease is a common fatal disease and is currently the number one killer of the global population. According to the World Health Organization report [1], cardiovascular disease kills 17.9 million people every year, accounting for about 32% of the world's deaths. The report also stated that heart disease and stroke are the leading causes of cardiovascular diseases, accounting for approximately 85% of deaths. Like a circulatory system disease, cardiovascular disease is caused by many factors, such as high blood pressure, smoking, diabetes, and lack of exercise.

So far, methods to reduce deaths from heart diseases have always been the focus of research, and studies have shown that about 90% of heart diseases can be prevented [2]. In addition, heart disease has the characteristics of early detection, early treatment, and early recovery. Therefore, early detection of this illness is the key to treatment. To obtain the patient's cardiovascular status, the hospital needs to collect specific physical values, such as static blood pressure, blood sugar, cholesterol, maximum heart rate, chest pain type, and electrocardiogram. However, traditional manual analysis of huge heart disease-related data has the disadvantages of misdiagnosis and is time-consuming. Artificial intelligence is widely used in prediction to solve this problem, among which machine learning (ML) and deep learning (DL) are the majority. These prediction models analyze a large amount of medical data to determine whether a patient has the disease and obtain more accurate prediction results than manual diagnosis.

This study combines machine learning with deep learning, applies LinearSVC and DNN technology, and proposes a new heart disease prediction model. The LinearSVC algorithm is applied to the feature selection module after data preprocessing. At the same time, we use Lasso as a penalty term to generate a sparse weight matrix, filter out a subset of features closely related to heart disease, and provide more reliable input for DNN. Furthermore, we compare several widely used weight initializers and finally choose the He initialization method since it can provide the best initial weight for the network. According to the results, the proposed model achieved accuracy, recall, and precision of 98.56%, 99.35%, and 97.84%.

The paper is structured as follows: Section 2 reviews the previous research on heart disease, Section 3 introduces the database we use and method analysis of our proposed model, followed by the detailed results of this research and the comparison with other algorithms in Section 4, and finally, Section 5 mentions a conclusion of this paper.

## 2. Literature Review

Researchers apply various data mining techniques to heart disease prediction methods. Amin et al. [3] used the UCI Cleveland database to confirm important features and mining techniques and finally used the UCI Statlog dataset for evaluation and verification. The research proposed 9 salient features from the 13 features of the original dataset and compared three data mining techniques: Vote, Naïve Bayes (NB), and Support Vector Machine (SVM). Among them, Vote has the best performance, and the accuracy is 87.41%. Similarly, Nalluri et al. [4] compared the performance of the XGBoost algorithm and the logistic regression (LR) method in predicting the value of Chronic Heart Disease (CHD). The results show that the accuracy of LR reaches 85.86%, which is better than XGBoost, which has an accuracy of 84.46%. Louridi et al. [5] used the UCI machine learning repository and compared three methods: SVM, k-Nearest Neighbor (kNN), and NB. Experiments show that the SVM with linear kernel has the best effect, with an accuracy of 86.8%. Shah et al. [6] used an existing dataset from the Cleveland database of the UCI Cardiology Patient Repository and considered 14 attributes. They compared four ML algorithms, namely, kNN, NB, DT, and random forest. The experimental results showed that kNN classification has the best effect (90.78%).

Decision tree (DT) also plays an essential role in the field of heart disease prediction. Kumar et al. [7] evaluated and analyzed three methods: NB, SVM, and DT, and the results showed that methods achieved 81.58%, 61.26%, and 90.79% accuracy. The effect of comparing DT is better than others. In a similar research, Pires et al. [8] compared a wealth of machine learning methods on neural networks, KNN, DT, SVM, combined nomenclature (CN2) rule inducer, and Stochastic Gradient Descent (SGD). The cross-validation results with different multiples show that DT and SVM have the best accuracy of 10-fold and 20-fold cross-validation (87.69%), and SGD has the best effect of 5-fold cross-validation (87.69%). There are also studies using mixed models to make predictions. Kavitha et al. [9] used random deep forest (RF), DT, and mixed model (RF; DT) on the UCI Cleveland dataset. The final result showed that the mixed model has the best effect, with an accuracy of 88.7%.

In addition, many new predictive models have also been proposed by researchers. Spencer et al. [10] combined feature selection technology with ML algorithm, and the created model combined chi-square feature selection and BayesNet algorithm to achieve an accuracy of 85%. Khan [11] proposed an improved deep convolutional neural network IoT framework. The framework is attached to a wearable detection device to detect the patient's blood pressure and electrocardiogram (ECG). Compared with the existing deep learning neural network and LR, this method has better performance (98.2%). Mohan et al. [12] combined RF with linear method (LM) and proposed a hybrid random forest (HRFLM) prediction model with a linear model. Experiments on the UCI Cleveland dataset showed that the accuracy of the classification model reached 88.7%, which is better than other classification methods. Magesh and Swarnalatha [13] adopted a cluster-based DT learning (CDTL) method. After feature processing, the CDTL-RF prediction accuracy can reach 89.30%, improving 12.60% compared to the non-CDTL method. Mehmood et al. [14] proposed a method called CardioHelp, which combines CNN with deep learning algorithms, involving the use of CNN for HF prediction and temporal model modeling at the earliest stage. Compared with other state-of-the-art methods, this method achieves the best performance, and its accuracy rate is 97%.

## 3. Materials and Methods

Data preprocessing, feature selection, and classification are the three most crucial parts of the heart disease prediction model. We carry out outlier processing and standardization on the dataset, ensuring all the data are well structured after the data preprocessing process. A feature selection process based on the LinearSVC algorithm is applied to choose valuable features. The selected feature subset is divided into the training set and test set at a ratio of 3 : 1; the former is fed into the deep neural network we built. Specifically, our deep neural network uses the he_normal initializer to construct the best initial weights to prevent gradients from exploding or vanishing and attain a better effect. Additionally, the effectiveness of the model is measured based on the test samples. The structure of our heart disease prediction model can be clearly seen in Figure 1.

### 3.1. Data Collection

There are many databases related to heart diseases, such as the Cleveland database and the heart disease database provided by the National Cardiovascular Disease Surveillance System. This paper uses a widely used heart disease dataset from Kaggle [15], composed of four databases: Cleveland, Hungary, Switzerland, and the VA Long Beach. The dataset has 14 attributes, and each attribute is set with a value. It contains 1025 patient records of different ages, of which 713 are male, and 312 are female. This dataset is a subset of [16]. The original dataset contains 76 attributes, but most scholars only use 14 of them, since other attributes have little effect on heart disease, such as time of exercise ECG reading and exercise protocol. The descriptions in this database are shown in Table 1.

### 3.2. Data Preprocessing

We choose the heart disease dataset publicly from Kaggle [15]. To ensure the stability and accuracy of the prediction model, it is essential to perform data analysis and preprocess before inputting them into the deep neural network. There are two main parts of data preprocessing: outlier removal and data standardization.

#### 3.2.1. Outlier Removal Process

Well-processed and structured data determines the effectiveness of the model largely. The raw dataset contains a sort of unreasonable values commonly, whose attributes are inconsistent with the whole. These abnormal values are named outliers. We analyze the heart disease dataset and apply the interquartile range (IQR) method to detect and remove outliers. It is worth mentioning that the physical indicators of healthy people are usually in a similar range, and the abnormality of specific biological indicators may be a reflection of diseases.

Therefore, the heart disease prediction model needs to alert some outliers instead of removing all of them thoughtlessly. This paper applied the IQR method to deal with the outliers of chol and trestbps columns since these two columns are generally normally distributed, but the boxplot shows that they both have apparent abnormalities that deviate from the normal range. IQR is a technique used to help detect outliers in data. It defines the difference between the third quartile and the first quartile as IQR [17], and then the lower and upper boundaries can be calculated by the following equations:

(1) $$\begin{array}{c} \text{IQR}=Q_{3}-Q_{1},\\ B_{l}=Q_{1}-1.5*\text{IQR},\\ B_{u}=Q_{3}+1.5*\text{IQR}. \end{array}$$

Now, the values outside the range of *B*_*l*_ ∼ *B*_*u*_ are recognized as outliers needed to be removed. After these outliers are filtered out, they can be abandoned from the dataset.  Figure 2 shows the changes in the boxplot before and after the outlier processing.

#### 3.2.2. Data Standardization Process

Data standardization aims to eliminate the differences between features so that subsequent models can learn weights wholeheartedly. Networks trained on standardized data usually produce better results [18]. Data standardization can convert the original data into normally distributed data without changing the initial data structure distribution. We use the StandardScaler method to standardize the data since all outliers are removed in the previous step and our data roughly obeys normal distribution. The conversion equation is as follows:

(2) $$\begin{array}{c} x^{*}=\frac{x-\mu }{\sigma }, \end{array}$$

where *u* is the mean of the training samples or zero if *with_mean* *=* *False* and *s* is the standard deviation of the training samples or one if *with_std* *=* *False*.

Standardization calculates the mean and variance of the data and converts the data with them. The standardization process can transform the data into a standard normal distribution suitable for the network behind it.

### 3.3. Feature Selection Based on an Embedded Method

Irrelative features often affect the model's training process, and some noise features even make the model deviate from the correct track. Feature selection chooses a subset of variables that can effectively describe the input data and ensure good prediction results [19]. Some feature selection methods are applied to reduce the influence of noise or irrelevant variables, roughly summarized into filter methods, wrapper methods, and embedded methods. However, the feature subset selected by the filter method has high redundancy, and the wrapper method has a high computational complexity because the evaluation of different feature subsets requires retraining and testing while the embedded method can efficiently select a subset with better performance. In this paper, the dataset we used has selected 14 attributes from 76 features in the original dataset. We use the penalty-based embedded feature selection method to verify these chosen features and try to pick the most related features based on them. Embedded feature selection integrates the feature selection process with the model training process. Instead of splitting the data into training and test sets, the two are completed in the same optimization process. The machine learning algorithm is used for training and obtains the weight coefficient of each feature, these weight coefficients often represent the importance of features to the model, and then the evaluation module selects the most contributing feature according to the value of the weight coefficient. The embedded feature selection method relies on model evaluation to complete feature selection.

Our embedded feature selection is based on the LinearSVC algorithm, which is applicable to this binary classification problem. We use L1 norm regularization [20] as a penalty term because it has good robustness and makes the coefficients sparse. The L1 regularization loss function is also called Lasso regression. It is expressed as follows:

(3) $$\begin{array}{c} \underset{w}{\min}\sum_{i=1}^{N}{\left(w^{T}x_{i}-y_{i}\right)}^{2}+\lambda w_{1}, \end{array}$$

where *w* represents the coefficient of the feature, *x* is the feature matrix, *y* is the target vector matrix, *n* is the number of samples, and *λ* represents the regularization strength.

The regularization can restrict the coefficient, and a sparse matrix can be obtained by using L1 regularization. The feature with a coefficient of 0 in the matrix can be regarded as inconsequential to the model, which will not affect the effectiveness of the model even if it is removed. Therefore, we can concentrate on the nonzero value features to achieve the purpose of feature selection. Through feature selection, we can reduce the number of features and select the most reliable feature subset.

### 3.4. Heart Disease Classification Using Deep Neural Networks

#### 3.4.1. Deep Neural Networks

A deep neural network is a deep learning framework, usually a feedforward neural network. In addition, the deep neural network is a discriminative model, which can be trained through the backpropagation algorithm [21].

After continuous research, the network has been widely used in speech recognition, cancer detection, and other fields and has outstanding performance. This is because deep neural networks can use statistical learning methods to extract high-level features from the input data.

The basic structure of DNN can be divided into three layers, namely, the input layer, hidden layer, and output layer. Unlike perceptrons, deep neural network structures have at least one hidden layer. Therefore, deep neural networks are sometimes called Multilayer Perceptrons (MLP). This change increases the depth and complexity of the model, improves the model's capabilities, and can use multiple activation functions. Each hidden layer of the network has interconnected neurons. The process of the deep neural network is that after the hidden layer extracts the input features, the classification result is finally obtained in the output layer. Our DNN network structure diagram is shown in Figure 3. We input the 12 features selected in the feature selection module into the DNN network. This network has 7 hidden layers and finally gets 2 outputs, corresponding to the scores belonging to each category.

#### 3.4.2. Loss and Activation Function

The heart disease prediction in this paper is essentially a binary classification problem. We use BinaryCrossentropy as a loss function to measure the quality of the model's prediction. BinaryCrossentropy is widely used in binary classification problems. To calculate the loss by BinaryCrossentropy, the following equation is used.

(4) $$\begin{array}{c} H_{p}\left(q\right)=-\frac{1}{N}\sum_{\text{i}=1}^{N}y_{\text{i}}\log\left(p\left(y_{i}\right)\right)+\left(1-y_{i}\right)\log\left(1-p\left(y_{i}\right)\right), \end{array}$$

where *y* is a binary label, and *p* (*y*) is the probability of belonging to the *y* label.

BinaryCrossentropy can measure the quality of classification since the process of reducing the loss can make the sample whose label equals 1 obtained a larger predicted probability of *p* (*y*). In contrast, the probability of the sample with 0 labels becomes smaller. The accuracy of the model can be significantly improved with the process of reducing loss.

The input layer and hidden layer of our deep neural network use the ReLU activation function, while the Sigmoid activation function is used in the output layer to map the output to the range of [0, 1] to adapt to the BinaryCrossentropy loss function. In addition, choosing Sigmoid instead of ReLU makes the output easier to control. The ReLU and Sigmoid functions are as follows:

(5) $$\begin{array}{c} \text{ReLu}\left(x\right)=\max\left(0,x\right),\\ \text{Sigmoid}\left(x\right)=\frac{1}{1+e^{-x}}. \end{array}$$

The output result obtained by Sigmoid can be regarded as the probability of belonging to the corresponding category. Therefore, we convert the data label into one-hot encoding. The one-hot encoding uses an N-bit status register to encode N states. The label is represented as a binary vector. In each code, only one bit is marked as 1, which represents a valid index, and the remaining bits are marked as 0. This encoding method converts the label into a convenient form for the network, which facilitates the calculation of the BinaryCrossentropy loss function.

#### 3.4.3. Application of Initializers

Deep neural networks usually need to learn an extremely complex nonlinear model, and different initializers often lead to distinctive convergence speeds and effects. If the weights of each layer are all initialized to 0 or 1, the neural network cannot learn important features during the backpropagation process, and it is challenging to update parameters. In addition, an excessively large initial value will cause exploding gradient, while an initial value that is too small will cause the vanishing gradient; both lead to a decline in the learning ability of the network. To solve the problems mentioned above, it is necessary to find a suitable weight initialization method, which needs to meet the following demands:

1. Avoid saturation of activation values of neurons in each layer
2. Avoid the activation value of each layer which becomes zero

However, the prevalent random normal method for weight initialization may cause network optimization to a dilemma. Once the random distribution is not properly generated, it may encounter a situation where the output value of the deep network is close to 0, resulting in the vanishing gradient. The basic idea of Xavier [22] initialization is that the activation value of each layer and the variance of the gradient remain consistent during the propagation process, avoid all output values tending to 0, and make each layer get effective feedback during backpropagation. However, Xavier initialization has an advantage over Tanh but is ineffective with the ReLU activation function. He initialization [23] divides by two based on Xavier, which can keep the variance unchanged and make sure half of the neurons in each layer are activated. Equation (6) states the Xavier method, and equation (7) states He initialization method.

(6) $$\begin{array}{c} w_{i}∼U\left(-\sqrt{\frac{6}{n_{i}+n_{i+1}}},\sqrt{\frac{6}{n_{i}+n_{i+1}}}\;\right), \end{array}$$

(7) $$\begin{array}{c} w_{i}∼\frac{\left[U\left(-\sqrt{6/n_{i}+n_{i+1}},\sqrt{6/n_{i}+n_{i+1}}\right)\right]}{2}. \end{array}$$

We compare some famous weight initialization methods, whose results are illustrated clearly in Section 4. Due to the advantages of the He initializer with the ReLU activation function, we employ this method in our network.

## 4. Results and Discussion

We employed the proposed method to predict heart disease and evaluated the results. The heart disease dataset was preprocessed through outlier removal and data standardization at the beginning, after which a feature selection module was applied, and the selected feature subset was fed into the deep neural network for training. We tried a wide range of network optimization algorithms to improve the effect and stability of the model.

We divided the data into a training and a test set at a ratio of 3 : 1, and 20% of the training data was partitioned for verification. The DNN network was trained and learned in the training set. We calculate the accuracy, recall, precision, and F1-score indicators to evaluate these results. Accuracy can describe the number of correct predictions over all of the predictions. Recall refers to the proportion of real positive cases that are correctly predicted positive, and precision denotes the proportion of predicted positive cases that are correctly real positives [24]; F1-score is a measure combining both precision and recall and can be regarded as the harmonic average of the two. The following equations present calculation of them:

(8) $$\begin{array}{c} \text{accuracy}=\frac{\text{TP}+\text{TN}}{\text{TP}+\text{TN}+\text{FP}+\text{FN}},\\ \text{recall}=\frac{\text{TP}}{\text{TP}+\text{FN}},\\ \text{precision}=\frac{\text{TP}}{\text{TP}+\text{FP}},\\ F1-\text{score}=\frac{2*\text{precision}*\text{recall}}{\text{precision}+\text{recall}} \end{array}$$

where TP is the true positive, FP denotes the false positive, TN denotes the true negative, and FN is the false negative.

In our experiment, the Adam optimizer was selected, which is a stochastic gradient-based optimization. The Adam optimizer only needs first-order gradients and is computationally efficient with only little memory. This method calculates the individual adaptive learning rate of different parameters by estimating the first and second moments of the gradient, which has advantages compared with other optimization methods [25]. In this experiment, the learning rate is 0.0001, and the number of iterations is 150. To ensure the reliability of the results, all of the statistics we mentioned in this paper are average results of 10 experiments. It shows that our average accuracy is 98.56%, recall reaches 99.35%, precision is 97.84%, and F1-score achieves 0.983.  Table 2 represents the detailed results and Figure 4 shows the confusion matrix of the predicted results of an experiment.

In addition, we use ROC and AUC to evaluate the performance of the model. Receiver operating characteristic curve (ROC) is a curve drawn based on a series of different boundary values with a true positive rate on the ordinate and a false positive rate on the abscissa [26]. AUC is the area under the ROC curve, which represents the probability of the calculated score of the positive sample higher than that of the negative sample when the samples are randomly selected, which can measure the pros and cons of the prediction model. Results show that the average AUC value of our model is 0.983 and the ROC curve of an experiment can be seen in Figure 5.

In the data preprocessing, we used the IQR method to remove the outliers of chol and trestbps and successfully normalized the dataset. In the feature selection module, we use an embedded feature selection method based on LinearSVC, using the L1 norm as a penalty term, and successfully picked 12 features that contribute to the model. The fbs feature with a score of 0 is removed in this module. See Table 3 for each feature score.

By using the He initialization method, our model obtained outstanding stability and accuracy as a consequence. We compare the neural network's performance using the He initialization method, RandomNormal method, and Xavier method. It is concluded that the He initialization shows superiority, the accuracy is 9.3% and 13.3% higher than the random and Xavier method, respectively, recall is 9.0% and 12.4% higher, respectively, precision is increased by 9.3% and 14.2%, and F1-score is increased in the number of 0.083 and 0.127. These results are demonstrated in detail in Figure 6.

Additionally, we found that batch normalization performed poorly in our model. We add batch normalization after the fully connected layer. The accuracy, recall, precision, and F1-score of the model change to 97.5%, 98.3%, 96.7%, and 0.98, respectively, which are decreased by 1.1%, 1.0%, 1.1%, and 0.003. Comparison results are illustrated in Figure 7. We conjecture this is because He initializer already gives the network good initial weights, so that each layer of the network has good input and output values, avoiding the vanishing and exploding gradients.

Furthermore, we compared our method with some published methods proposed by other scholars. For example, Ramprakash et al. [27] used the combination of the PCA feature extraction method and DNN to get a classification with high accuracy, but the recall only reached 97%. The specific comparison results are shown in Table 4.

## 5. Conclusions

In this paper, we propose a heart disease prediction algorithm based on DNN combined with LinearSVC embedded feature selection method. Through the IQR method, the outliers in the dataset are successfully removed and all data are standardized to obtain reliable input. In addition, the optimal feature subset is selected in the feature selection module based on the LinearSVC algorithm and L1 norm. A total of 12 most-relative features are selected and input into the subsequent DNN network. To enhance the network's performance, we compare three weight initialization methods including the He_normal, random_normal, and Xavier, concluding that He initialization method acquires the best results in this heart disease prediction model. Meanwhile, we find that the batch normalization layer is not suitable for this method, attaining lower scores in every indicator. In this two-classification problem, we choose BinaryCrossentropy as the loss function and Sigmoid as the activation function of the output layer to map the output to the range of [0, 1]. The experimental results show that a high-accuracy prediction model for heart disease is realized. The accuracy of our proposed method reaches 98.56%, recall is 99.35%, precision is 97.84%, and F1-score achieves 0.983, with an AUC score of 0.983, proving that this feature selection method and deep neural network are feasible and reliable in predicting heart disease. In the future, we will continue to adjust the depth and parameters of the DNN to enhance the stability of the model as well as research other deep learning optimization techniques to obtain better performance [30].

## Figures and Tables

**Figure 1:** Proposed heart disease prediction system structure.

**Figure 2:** The changes of boxplot before and after the outlier removal using IQR. (a) Raw data. (b) Results of outlier removal.

**Figure 3:** The structure of our deep neural network.

**Figure 4:** Confusion matrix on test data.

**Figure 5:** ROC curve and AUC of the proposed algorithms.

**Figure 6:** Results of different initializers.

**Figure 7:** Comparison of results using batch normalization layer.

**Table 1:** Description of features.

SN	Attribute	Description
1	age	Age in years
2	sex	1 = male; 0 = female
3	cp	Chest pain type
4	trestbps	Resting blood pressure (in mm Hg on admission to the hospital)
5	chol	Serum cholesterol in mg/dl
6	fbs	Fasting blood sugar >120 mg/dl (1 = true; 0 = false)
7	restecg	Resting electrocardiographic results
8	thalach	Maximum heart rate achieved
9	exang	Exercise-induced angina (1 = yes; 0 = no)
10	oldpeak	ST depression induced by exercise relative to rest
11	slope	The slope of the peak exercise ST segment
12	ca	Number of major vessels (0–3) colored by fluoroscopy
13	thal	1 = normal; 2 = fixed defect; 3 = reversible defect
14	target	1 = disease; 2 = no disease

**Table 2:** Results of the proposed method.

	Class 0 (%)	Class 1 (%)
Accuracy	98.56	98.56
Recall	97.84	99.35
Precision	99.35	97.84

**Table 3:** Importance value of features.

SN	Attribute	Importance value
1	age	−0.00144
2	sex	−0.56535
3	cp	0.288000
4	trestbps	−0.005696
5	chol	−0.001637
6	fbs	0.0
7	restecg	0.1190487
8	thalach	0.0079078
9	exang	−0.332790
10	oldpeak	−0.199450
11	slope	0.1589541
12	ca	−0.252994
13	thal	−0.2927249

**Table 4:** Comparison of classification performance of the proposed method with others.

Authors	Methods	Accuracy (%)	Recall (%)	Precision (%)
Ramprakash et al. [27]	*χ* ^2^-DNN	94.0	93.00	—
Gao et al. [28]	Bagging ensemble method with decision tree	98.6	99.0	97.8
Gao et al. [28]	PCA + decision tree	99.0	97.0	98.0
Ali et al. [29]	MLP	97.95	98	98
Proposed	LinearSVC + DNN	**98.56**	**99.35**	**97.84**

## Data Availability

The heart disease dataset used to support the findings of this study is available at https://www.kaggle.com/johnsmith88/heart-disease-dataset.
